The article "Valproic Acid Inhibits Glioma and Its Mechanisms" was published in 2022. Journal: J Healthc Eng.

# Valproic Acid Inhibits Glioma and Its Mechanisms

**DOI:** 10.1155/2022/4985781

**Published:** 2022-02-10

**Authors:** Zhao-Yu Yang, Xiao-Hong Wang

**Affiliations:** ^1^Department of Neurosurgery, Dongying People's Hospital, Dongying 257091, Shandong, China; ^2^Department of Rehabilitation Medicine, Dongying People's Hospital, Dongying 257091, Shandong, China

## Abstract

Glioma is one of the most common intracranial tumors worldwide, and metastasis and chemoresistance remain a challenge in glioma treatment. This study aims to investigate the effect of sodium valproate on the invasion and metastasis of glioma cells and its mechanism. Glioma cell lines were stimulated with VPA at different concentrations and for different durations of action. U87 glioma cells were transfected with Smad4 plasmid and small interfering RNA, and the changes of EMT-related protein indexes in U87 cells after up- or downregulation of Smad4 were detected by Western blotting. Immunohistochemistry was used to detect the differences in the expression of Smad4, TIF1-*γ*, and TGF-*β* proteins in 39 glioma clinical specimens from the Department of Pathology of our hospital. Based on the regulation of EMT-related transcription factors by VPA, our study indicates that VPA inhibits the EMT process of glioma by altering the expression level of Smad4, which is induced by TGF-*β*1 to form a Smad3/4 complex, thus inducing the EMT process of the tumor and acting as an antitumor target to inhibit the invasive ability of glioma cells. Sodium valproate inhibits glioma invasion and metastasis through the regulation of Smad4 expression.

## 1. Introduction

Glioma is one of the most common intracranial tumors worldwide, and metastasis and chemoresistance remain a challenge in glioma treatment [1]. Epithelial-mesenchymal transition (EMT), a pathophysiologic process of conversion of epidermal cells to mesothelial cells in tissues, plays a very important role in the invasion and metastasis of tumors to adjacent and distant tissues and organs [2, 3]. During EMT, epidermal cells lose their cell polarity and cell-to-cell junctions and then acquire the characteristics of mesothelial cells, giving tumor cells a strong ability to invade and metastasize to distant organs and tissues. This process is caused by multiple complexes and growth factors in the tumor microenvironment, and TGF-*β* is one such factor that has both facilitating and inhibiting roles in the process of tumor invasion and metastasis. Studies have focused on the important role of TGF-*β* in different stages of tumorigenesis and EMT, but its role in the initial response to EMT remains unclear [4, 5]. TGF-*β* plays a tumor suppressor role in the early stage of tumor and a tumor promoter role in the late stage of tumor. Through both classical and nonclassical pathways of the TGF-*β* signaling pathway, TGF-*β* factors play a potentially inducible role in the formation of EMT, and Smad4 protein can serve as an independent factor in the prognosis of renal tumor patients. Histone acetylation and deacetylation are mechanisms by which histones are epigenetically modified to regulate gene expression [6, 7]. Histone acetyltransferases and deacetylases play an important role in the silencing and activation of oncogene expression, along with histone acetylation and deacetylation.

The article "Valproic Acid Inhibits Glioma and Its Mechanisms" was published in 2022. Journal: J Healthc Eng.

Valproate sodium (VPA) is a short-chain fatty acid that has been used for decades as a traditional classical antiepileptic drug and has been shown to be an HDAC inhibitor (HDACI) [8], which has been shown to regulate tumor cell differentiation and apoptosis in acute myeloid leukemia (AML) cancer [9]. The basic process of EMT is also an important step in the development of invasive metastasis in gliomas. In rectal cancer studies, the absence of E calcium-linked protein is also an essential feature of EMT in colon cancer cells. The role of VPA in antitumorigenesis is gaining more and more attention from researchers. Overexpression of HDACs often leads to dysfunctional cell differentiation, uncontrolled cell proliferation, and promotion of tumorigenesis and invasion; VPA has been proven to inhibit HDACs and has antitumor effects in prostate, colon, liver, cervical, lung, and ovarian cancers. In addition, VPA can also regulate the tumor cell cycle and the autophagy ability of prostate cancer cells [10]. Previous studies have shown that, during the process of EMT, tumor cells lose the polarity of epidermal cells and acquire the characteristics of mesothelial cells, intercellular junction properties are lost, the intercellular skeletal structure is reorganized, cells gain significant mobile invasive capacity, and tumor cell invasion and metastasis are enhanced.

In this study, the experimental results showed that the ability of VPA to inhibit tumor invasion and metastasis at different doses was dose-dependent and was accompanied by changes in the expression of Smad4 protein and EMT parameters. In glioma cancer, Smad4 protein was differentially expressed in different pathological samples, which further confirmed the key role of Smad4 in tumor invasion and metastasis. This study further revealed the inhibitory effect of VPA on tumor invasion and metastasis in different cell lines of glioma cancer and the possible relationship between VPA, Smad4, and EMT.

## 2. Materials and Methods

### 2.1. Cell Lines and Reagents

Human glioma SHG44 and U87 cell lines were purchased from the Institute of Cell Research, Chinese Academy of Sciences. Sodium valproate was purchased from Sigma, USA; all primary antibodies and horseradish peroxidase goat anti-mouse and anti-rabbit secondary antibodies were purchased from Santa, USA; fetal bovine serum and DMEM culture broth were purchased from Hyclone, USA; the complete protein extraction kit was purchased from Beijing Sulabal Biotechnology Co. Ltd.; Smad4 and GAPDH antibodies were purchased from Santa Cruz Corporation, USA; and Lipo2000 was purchased from Shanghai Biyuntian Biotechnology Co. Thirty-nine patients with glioma who had not received preoperative radiotherapy or chemotherapy from January to December 2019 were collected from the Department of Neurosurgery of our hospital. Their tumor tissues and paraneoplastic tissues (tissue in the penumbra removed during surgery, approximately 0.5 cm from the tumor tissue) were taken. All glioma tissues and normal tissues were confirmed by pathological examination and approved by the ethics committee of our hospital before collection. The tissues were removed and placed in liquid nitrogen for backup. Inclusion criteria were low-grade glioma and primary high-grade glioma with tumor sites limited to the lobes of the brain, no other underlying disease (diabetes, hypertension, heart disease, etc.), good preoperative neurological status, and no other treatment for glioma such as radiotherapy or chemotherapy before surgery. Exclusion criteria were diffuse infiltrative growth of glioma tissue in the dominant hemisphere, focal invasion of both hemispheres, poor preoperative neurological status, and malignant glioma deep in the brain or in the brainstem.

The article "Valproic Acid Inhibits Glioma and Its Mechanisms" was published in 2022. Journal: J Healthc Eng.

### 2.2. Transwell Cell Assay for Glioma Cell Invasion and Metastatic Capacity

After the intervention with sodium valproate, 0.2 ml of glioma cells was taken into the upper chamber of Transwell, 0.5 ml of DMEM containing 10% fetal bovine serum was added into the lower chamber, and the cells were incubated for 4 h. The cells were removed from the incubator for 24 h, swabbed with cotton swabs, washed with PBS, and fixed with formaldehyde for 15 min.

### 2.3. Western Blotting for the Expression of Cell Cycle and Apoptosis-Related Proteins

After grouping, collect the cells in a centrifuge tube and extract the protein using a protein kit. Each well was filled with 20 *μ*g of the sample. 10% to 12% of the sample was used for the extraction of protein. The proteins were separated by SDS-PAGE and transferred to nitrocellulose membranes by semidry electrotransfer. After 1.5 h of confinement of skim milk (5%), TBST was washed 5 times (5 min/time). Add the corresponding monoclonal antibody (dilution ratio 1 : 2 000) and incubate overnight at 4°C with shaking. The corresponding primary antibody was recovered, washed 5 times (5 min/time) with TBST, added to the corresponding secondary antibodies (HRP-labeled goat anti-rabbit and anti-mouse IgG), incubated for 1.5 h at room temperature in a shaking bed, washed 5 times (5 min/time) with TBST, developed using ECL chemiluminescence developer, and then photographed by the chemiluminescence imaging system. The *α*-tubulin was selected by an internal reference and analyzed by grayscale using ImageJ 1.42q software.

The article "Valproic Acid Inhibits Glioma and Its Mechanisms" was published in 2022. Journal: J Healthc Eng.

### 2.4. Immunohistochemical Detection of Smad4, TIF1-*γ*, and TGF-*β* Protein Expression in Glioma and Nonglioma Tissues

The carcinoma and paraneoplastic tissue specimens were fixed in 10% neutral formaldehyde solution for 24 h. The specimens were then embedded in paraffin and sectioned. The sections were immersed in hematoxylin solution for 35 min and then stained with alkaline nuclear stain. Acid-alcohol decolorization was performed, and tap water was used for bluing. Then, tissue specimens were washed and dehydrated with gradient ethanol step by step, and it was made transparent with xylene and fixed with rubber seal. The sections were dewaxed, the antigens were repaired with citric acid buffer at high temperature and high pressure, and then 50 *μ*l of 3% H2O2 was added and incubated at room temperature for 10 min. 50 *μ*l of primary antigen was added, 50 *μ*l of secondary antigen was added, 50 *μ*l of PBS was washed three times, and then 50 *μ*l of goat serum sealing solution was added and incubated at 37°C for 20 min. Wash the sections with PBS 3 times, add 100 *μ*l of DAB solution for color development, and terminate the development with purified water. Smad4, TIF1-*γ*, and TGF-*β* were positively expressed in the cytoplasm or nucleus and appeared as brownish-yellow granules. Five high-magnification fields were randomly selected, and 200 cells were counted in each field. Scoring by staining intensity was as follows: 0 points, no staining; 1 point, weak staining; 2 points, moderate staining; 3 points, dark staining. Score according to the percentage of positive cells was as follows: 0 points, the percentage of positive cells with staining ≤5%; 1 point, >5%∼25%; 2 points, >25%∼50%; 3 points, >50%. Multiplying the staining intensity score and the positive cell number percentage score gave the positive coefficient: 0 and 1 points were determined as (−), 2 and 3 points were determined as (+), 4 to 6 points were determined as (++), and 9 points were determined as (+++).

### 2.5. Statistical Processing

SPSS19.0 was used to analyze the mean ± standard deviation for measurement data and *t*-test or ANOVA for comparison.

The article "Valproic Acid Inhibits Glioma and Its Mechanisms" was published in 2022. Journal: J Healthc Eng.

## 3. Results

### 3.1. Expression of Smad4 Protein and EMT-Related Markers in Glioma Cells with Different Invasive Capacities

Smad4 and EMT-related proteins were differentially expressed in glioma cells with different invasive capacities. In SHG44, U87, and HEB, Smad4 mRNA and protein levels were significantly higher in U87 cells than in SHG44 cells and normal brain glial cells (HEB), whereas the expression of E-cadherin was lower (Figure 1). This result showed that Smad4 levels were significantly higher in highly invasive cells than in low-invasive cells and normal cells and that there was a potential link between Smad4 protein and cell invasive capacity.

### 3.2. VPA Inhibits Glioma Cell Invasion and Metastasis

The invasive metastatic ability of U87 and SHG44 tumor cells decreased significantly with increasing drug concentrations, and the low dose of VPA had only a limited inhibitory effect, but the relatively high dose of VPA had a significant inhibitory effect (*p* < 0.05) (Figures 2(a) and 2(b)). Moreover, the morphology of the VPA-treated cells changed from ellipsoidal to more rod-shaped (Figure 2(c)).

### 3.3. VPA Alters the Expression of EMT-Related Indicators

In glioma SHG44 and U87 cell lines, we used immunoblotting to analyze the expression changes of EMT-related index proteins and Smad4 protein after VPA treatment. Vimentin was downregulated, whereas E-cadherin expression levels were shown to be upregulated (Figures 3(a) and 3(b)). From the results of real-time PCR, we further clarified that, at the mRNA level, Smad4, N-cadherin, and VPA have an impact on the EMT process in both glioma cell lines after treatment with different VPA doses (control, 1.2, 2.4, and 5 mmol/1) and for different times (0, 12, 24, and 48 hours). The same trend of decreasing vimentin expression and increasing E-cadherin expression existed (Figure 3(c)). This change in protein level was observed in the mode of treatment with different doses of VPA (control, 1.2, 2.4, and 5 mmol/l) and at different time points (0, 12, 24, and 48 hours) with the same VPA concentration, which more fully demonstrates the effect of VPA on the EMT process.

### 3.4. The Inhibitory Effect of VPA on the EMT Process Is Achieved by Smad4 Expression

In U87 cells, we transfected Smad4 cDNA plasmid and shRNA interfering plasmid to interfere with the expression of Smad4, and the immunoprotein blotting results confirmed that the expression of Sraad4 protein was significantly increased in the overexpression group and decreased in the low expression group. The transfected cells were also treated with VPA (2.4 mmol/l). The immunoprotein blotting results showed that the expression of N-cadherin and vimentin was increased in the cells overexpressing Smad4, while the expression of E-cadherin was decreased in the cells overexpressing Smad4 (Figure 4(a)). In cells with low expression of Smad4, the expression of N-cadherin and vimentin was decreased, while E-cadherin expression was increased. When VPA treatment was administered, we found that there was no significant trend in the expression of E-cadherin and N-cadherin in the VPA-treated and control groups (Figure 4(b)), indicating the presence of Smad4 protein. This indicates that the presence of Smad4 protein plays a crucial role in the inhibition of the EMT process by VPA.

The article "Valproic Acid Inhibits Glioma and Its Mechanisms" was published in 2022. Journal: J Healthc Eng.

### 3.5. Expression of Smad4, TIF1-*γ*, and TGF-*β* in Glioma Samples

To better understand the role of Smad4 protein in the TGF-*β* pathway, we analyzed the expression of Smad4, TIF1-*γ*, and TGF-*β* proteins in 39 glioma specimens from the Department of Pathology of our hospital using immunohistochemistry. According to the pathological results, among the 39 samples, 8 cases (20.5%) had G I stage, 24 cases (61.5%) had G II stage, and 7 cases (18%) had G III stage. Five cases (12.8%) had high expression of TGF-P (Figure 5(a)), and 21 cases (53.8%) had low expression (Figure 5(b)). The expression of Smad4 in the nucleus and cytoplasm was high in 6 cases (15.4%) (Figure 5(c)) and low in 21 cases (53.8%) (Figure 5(d)), and the expression of TIF1-*γ* was high in 5 cases (12.8%) (Figure 5(e)) and low in 19 cases (48.7%) (Figure 5(f)). Based on immunohistochemical and statistical analysis, we found that Smad4 expression was associated with higher tumor grade (*p*=0.048), and TIF1-*γ* expression was also associated with tumor grade (*p*=0.014), with lower protein expression being associated with lower tumor grade (Tables 1 and 2). However, there was no significant association between Smad4, TIF1-*γ*, and TGF-*β* proteins as independent prognostic factors and patient age, tumor size, PTNM stage, and tumor-associated survival.

## 4. Discussion

Previous studies have shown that, during the process of EMT, tumor cells lose the polarity of epidermal cells and acquire the characteristics of mesothelial cells, intercellular junction properties are lost, the intercellular skeletal structure is reorganized, cells gain significant mobile invasive capacity, and tumor cell invasion and metastasis are enhanced [2]. The basic process of EMT is also an important step in the development of invasive metastasis in gliomas. In rectal cancer studies, the absence of E calcium-linked protein is also an essential feature of EMT in colon cancer cells [11]. The early metastasis of tumor cells is an important clinical challenge for glioma patients. Histone deacetylase inhibitors (HDACi) are considered chemotherapeutic agents with potential antitumor properties [12]. Preclinical studies have found that different modifications and epigenetic alterations of histones lead to altered cellular activity and inhibition of tumor growth, differentiation, and apoptosis, which are important in the invasion and metastasis of tumor cells. DNA methylation and mutation of some histone sites are associated with tumor invasion and metastasis. HDACi inhibitors such as Trichostatin A (TSA) and sodium butyrate (NaB) exert their effects on the inhibition of tumor stem cells (CSCs) in squamous cell carcinoma by regulating the acetylation of nonhistone proteins, thereby affecting several transcription factors including *p*53, STAT3, and other transcription factors, and can enhance the sensitivity of tumor cells to drug therapy [13–15]. In addition, the inhibition of tumor cells by HDACi drugs such as MS-275 and Vorinostat has also been demonstrated in a variety of tumors.

The article "Valproic Acid Inhibits Glioma and Its Mechanisms" was published in 2022. Journal: J Healthc Eng.

It has been shown that VPA inhibits the growth of prostate cancer cells by inhibiting the EMT process in prostate cancer cells. The mechanism is that VPA affects the function of Smad4 protein in the TGF-*β* pathway, resulting in decreased protein expression and monoubiquitination of Smad4 protein, leading to a decrease in Sraad4 nucleation and intracellular Sraad4 protein [16]. In vitro and in vivo experiments have demonstrated that VPA has the ability to inhibit growth and promote apoptosis in ovarian cancer cells and to alter the cell cycle in ovarian cancer cells, resulting in a decrease in the S phase, an increase in the G1 phase, an increase in the E calnexin expression, and a decrease in the metalloproteinase 9 (MMP9) expression [17]. HDACi has been used in glioma therapeutic studies, and the combination of mTOR inhibitors and HDACi can inhibit the mTOR signaling pathway, thereby suppressing oncogene expression, reducing protein synthesis, leading to cell cycle arrest, and thus affecting tumor cells' HDACi, which has an invasive capacity and has entered clinical phase III trials in metastatic renal cell carcinoma. HDACi, as a deacetylase inhibitor, can alter the expression of relevant genes by regulating the acetylation modification of histones [18]. Similar effects have also been found in thyroid cancer cells, as well as in clinical research work on adenoid cystic carcinoma [19]. As an old drug, new effects were discovered, as VPA not only inhibits tumor growth and metastasis but also induces differentiation and apoptosis in tumor cells in vitro and in vivo. In our experiments, VPA reversed the EMT process in glioma and affected EMT index-related proteins in U87 and SHG44 cells, which provide new targets for the treatment of glioma.

The article "Valproic Acid Inhibits Glioma and Its Mechanisms" was published in 2022. Journal: J Healthc Eng.

Numerous studies have demonstrated that the TGF-*β* pathway has a role in inducing the EMT process and regulating tumorigenesis. Smad4 plays an important role in the TGF-*β* pathway-regulated EMT process. Smad proteins are divided into three parts, receptor Smads (R-Smads), chaperone Smads (Co-Smad), and inhibitor Smads (I-Smads). tGF-*β* phosphorylates Smad2/3 by causing phosphorylation of Smad2/3 in the cytoplasm, which results in the phosphorylation of Smad4 and Smad4. Smad2 and S/mad3 enter the nucleus to form a complex with Smad4, which binds to the enhancer region of the gene (SBE) and regulates the expression of downstream gene proteins. Understanding the TGF-*β* regulatory process will help us to better explain the key role of Smad4 protein in the EMT process, based on previous studies on the link between the TGF-*β* pathway and Smad4. Therefore, it was necessary to verify the relationship between Smad4 and EMT in glioma cells to confirm the role of this protein in the invasion and metastasis of tumor cells. In our in vitro experiments, U87 cells were transfected with the Smad4 shRNA plasmid, which decreased the expression of Smad4 protein. The difference in properties between the mesothelium and the epidermis is determined by the function of E and N calnexin, and these factor proteins can be used as targets for cancer therapy. In our study, low expression of Smad4 in glioma cells produced a similar effect to that of VPA, with inhibition of tumor invasion and metastasis. The calmodulin/*E* calmodulin transcriptional pathway affects the invasive metastatic process of tumor cells. Overall, these findings contribute to our new understanding of the critical role of Smad4 in the TGF-*β* pathway induction of EMT, but we still do not fully understand what regulates the transformation of TGF-*β* from early tumor suppression to late tumor promotion and the function of Smad4 protein in this process has not been fully elucidated. Some studies have reported that Smad4 protein can act as an independent prognostic factor, and the expression of Smad4 in the nucleus is strongly correlated with tumor size, nuclear grade, pTNM, and tumor invasion progression. After reducing the expression of Smad4 protein, the expression of N calnexin was significantly decreased, and the expression of E calnexin was significantly increased. By transfecting U87 cells with Smad4 overexpression plasmid, we upregulated Smad4 protein expression and found that this resulted in a decrease in E calnexin expression and an increase in N calnexin expression in the cells. In tumor cells, E and N calnexin significantly regulate the invasion and metastasis of tumor cells and are two essential factor proteins that influence cell signaling and cell physical connectivity. In breast cancer, tumor cells often secrete excess TGF-*β* protein, forming Smad3/Smad4 complexes in the nucleus, which increases the expression of SLUG protein and promotes tumor invasion, and knockdown of Smad3 protein reduces tumor invasion and metastasis. SBEs bind to the enhancer subdomain of N calnexin and regulate its expression. Interestingly, it has also been found in hepatoma cells that high levels of Smad4 expression are associated with poorer prognosis after surgery, and knockdown of Smad4 protein significantly inhibits colony formation and the migratory ability of hepatocytes, whereas binding of nuclear Smad4 protein to phosphorylated Smad2/3 promotes invasive metastasis in hepatoma patients.

The article "Valproic Acid Inhibits Glioma and Its Mechanisms" was published in 2022. Journal: J Healthc Eng.

## 5. Conclusion

Our study confirmed the inhibitory effect of VPA on the EMT process and further investigated the role of Smd4 protein in this inhibitory process. In addition, based on our previous studies on the effect of VPA on Smad4 monoubiquitination leading to its nucleation and on the role of TIF1-*γ* as a monoubiquitination enzyme in the regulation of Smad4 monoubiquitination and its entry into and exit from the nucleus, it is clear that VPA has no role in the regulation of EMT. The results of our study, coupled with our findings on the correlation between Sniad4 and TIF1-*γ* expression and tumor stage in clinicopathological samples, suggest that later studies should also focus on the relationship between TIF1-*γ* and ubiquitinated Smad4 protein. In the future, our research direction should focus on the mechanism of action. Our experiment has many limitations, and more experimental cases are needed to verify our conclusions. Overall, our study further elucidates the role of Smad4 in tumor invasion and metastasis, discusses the different mechanisms of tumor invasion and metastasis and the key regulatory role of Sniad4 protein in the EMT process, and provides a prospect for using Smad4 as a new clinical index in the future.

## Figures and Tables

**Figure 1:** Expression of Smad4 and EMT-related proteins in different glioma cell lines and normal brain glial cells. (a) Western blotting technique was used to detect the differences in the expression levels of Smad4 protein and EMT-related index proteins in different cell lines U87, SHG44, and HEB. (b) Differences in mRNA levels of Smad4 and EMT-related indicators in U87, SHG44, and HEB were detected by RT-PCR in different cell lines (^*∗*^*p* < 0.05).

**Figure 2:** (a) Changes in invasive capacity (200x) and statistics of average perforated cells of glioma U87 cells at different concentrations of VPA (1.2 mmol/l, 2.4 mmol/l, and 5 mmol/l). (b) Statistics of the invasion ability of glioma SHG44 cells at different concentrations of VPA (1.2 mmol/l, 2.4 mmol/l, and 5 mmol/l) (200x) and the average permeabilized cells. (c) Different morphological and quantitative alterations of U87 cells after VPA quantification (top row: 0 mmol/1, 1.2 mmol/l, 2.4 mmol/l, and 5 mmol/l) and aging (bottom row: 0 h, 12 h, 24, and 48 h).

The article "Valproic Acid Inhibits Glioma and Its Mechanisms" was published in 2022. Journal: J Healthc Eng.

**Figure 3:** Smad4 and EMT-related proteins are expressed in VPA-treated glioma cells. (a) Effect of VPA on the expression of Smad4 and EMT-related proteins in glioma SHG44 cells by aging (0 h, 12 h, 24, and 48 h) and quantification (0 mmol/l, 1.2 mmol/l, 2.4 mmol/l, and 5 mmol/l). (b) Effect of VPA on the expression of Smad4 and EMT-related proteins in glioma U87 cells by aging (0 h, 12 h, 24, and 48 h) and quantification (0 mmol/l, 1.2 mmol/l, 2.4 mmol/l, and 5 mmol/l). (c) The effects of VPA on the expression of Smad4, N-cadherin, E-cadherin mRNA in glioma cells SHG44 and U87 were detected by RT-PCR after time-effect (0 h, 12 h, 24, and 48 h) and dose-effect (0 mmol/l, 1.2 mmol/l, 2.4 mmol/l, and 5 mmol/l) of VPA.

**Figure 4:** Western blot analysis of the expression of U87-related proteins after different treatments. (a) Overexpression of Smad4 (0E-Smad4) and altered expression of the EMT-related proteins, E-cadherin, N-cadherin, and vimentin after VPA treatment. (b) Low expression of Smad4 (KD-Smad4) and altered expression of the EMT-related proteins, E-cadherin, N-cadherin, and vimentin after VPA treatment (^*∗*^*p* < 0.05, compared to blank controls).

**Figure 5:** Immunohistochemical results. High expression (a) and low expression (b) of TGF-*β*1 in tumor cells, low expression (c) and high expression (d) of Smad4 outside the nuclear nucleus of tumor cells, and high expression (e) and low expression (f) of TIF1-*γ* protein in tumor cells.

**Table 1:** Expression of Smad4 in 39 clinical samples.

	Low expression	Medium expression	High expression	*p*
GI	3	4	1	*p*=0.048
GII	15	8	I	
GIII	2	1	4	
	20	13	6	

**Table 2:** Expression of TIF1-*γ* in 39 clinical samples.

	Low expression	Medium expression	High expression	*p*
Installment GI	5	3	0	*p*=0.014
GII	13	10	1	
GIII	1	2	4	
	19	15	5	

## Data Availability

The datasets used and/or analyzed during the current study are available from the corresponding author upon reasonable request.

## References

[1] Ludwig K., Kornblum H. I. (2017). Molecular markers in glioma. *Journal of Neuro-Oncology*.

[2] Lamouille S., Xu J., Derynck R. (2014). Molecular mechanisms of epithelial-mesenchymal transition. *Nature Reviews Molecular Cell Biology*.

The article "Valproic Acid Inhibits Glioma and Its Mechanisms" was published in 2022. Journal: J Healthc Eng.

[3] Kalluri R., Weinberg R. A. (2009). The basics of epithelial-mesenchymal transition. *Journal of Clinical Investigation*.

[4] Colak S., Ten Dijke P. (2017). Targeting TGF-*β* signaling in cancer. *Trends in Cancer*.

[5] Xie F., Ling L., van Dam H., Zhou F., Zhang L. (2018). TGF-*β* signaling in cancer metastasis. *Acta Biochimica et Biophysica Sinica*.

[6] Guo P., Chen W., Li H., Li M., Li L. (2018). The histone acetylation modifications of breast cancer and their therapeutic implications. *Pathology and Oncology Research*.

[7] Benton C. B., Fiskus W., Bhalla K. N. (2017). Targeting histone acetylation. *The Cancer Journal*.

[8] Amiri-Nikpour M. R., Nazarbaghi S., Eftekhari P. (2018). Sodium valproate compared to phenytoin in treatment of status epilepticus. *Brain Behav*.

[9] Goodyear O., Agathanggelou A., Novitzky-Basso I. (2010). Induction of a CD8+ T-cell response to the MAGE cancer testis antigen by combined treatment with azacitidine and sodium valproate in patients with acute myeloid leukemia and myelodysplasia. *Blood*.

[10] Gavrilov V., Leibovich Y., Ariad S., Lavrenkov K., Shany S. (2010). A combined pretreatment of 1,25-dihydroxyvitamin D3 and sodium valproate enhances the damaging effect of ionizing radiation on prostate cancer cells. *The Journal of Steroid Biochemistry and Molecular Biology*.

[11] Chen H.-N., Yuan K., Xie N. (2016). PDLIM1 stabilizes the E-cadherin/*β*-catenin complex to prevent epithelial-mesenchymal transition and metastatic potential of colorectal cancer cells. *Cancer Research*.

[12] Beier U. H., Akimova T., Liu Y., Wang L., Hancock W. W. (2011). Histone/protein deacetylases control Foxp3 expression and the heat shock response of T-regulatory cells. *Current Opinion in Immunology*.

[13] Suraweera A., O’Byrne K. J., Richard D. J. (2018). Combination therapy with histone deacetylase inhibitors (HDACi) for the treatment of cancer: achieving the full therapeutic potential of HDACi. *Frontiers in Oncology*.

[14] Bose P., Verstovsek S. (2016). Investigational histone deacetylase inhibitors (HDACi) in myeloproliferative neoplasms. *Expert Opinion on Investigational Drugs*.

[15] Rivera-Del Valle N., Cheng T., Irwin M. E., Donnella H., Singh M. M., Chandra J. (2018). Combinatorial effects of histone deacetylase inhibitors (HDACi), vorinostat and entinostat, and adaphostin are characterized by distinct redox alterations. *Cancer Chemotherapy and Pharmacology*.

[16] Lan X., Lu G., Yuan C. (2016). Valproic acid (VPA) inhibits the epithelial-mesenchymal transition in prostate carcinoma via the dual suppression of SMAD4. *Journal of Cancer Research and Clinical Oncology*.

The article "Valproic Acid Inhibits Glioma and Its Mechanisms" was published in 2022. Journal: J Healthc Eng.

[17] Shan Z., Feng-Nian R., Jie G., Ting Z. (2012). Effects of valproic acid on proliferation, apoptosis, angiogenesis and metastasis of ovarian cancer in vitro and in vivo. *Asian Pacific Journal of Cancer Prevention*.

[18] Lee J. H., Choy M. L., Ngo L., Foster S. S., Marks P. A. (2010). Histone deacetylase inhibitor induces DNA damage, which normal but not transformed cells can repair. *Proceedings of the National Academy of Sciences*.

[19] Xu Y., Xu D., Zhu S. J. (2015). Induction of apoptosis and autophagy in metastatic thyroid cancer cells by valproic acid (VPA). *International Journal of Clinical and Experimental Pathology*.

